The article "Design of Machine Learning Algorithm for Tourism Demand Prediction" was published in 2022. Journal: Comput Math Methods Med.

# Design of Machine Learning Algorithm for Tourism Demand Prediction

**DOI:** 10.1155/2022/6352381

**Published:** 2022-06-08

**Authors:** Nan Yu, Jiaping Chen

**Affiliations:** ^1^School of Tourism, Yellow River Conservancy Technical Institute, Kaifeng, Henan 475000, China; ^2^School of Tourism, Henan Vocational & Technical College, Zhengzhou, Henan 450000, China

## Abstract

Unused hotel rooms, unused event tickets, and unsold items are all examples of wasted expenses and earnings. Governments require accurate tourism demand forecasting in order to make informed decisions on topics such as infrastructure development and lodging site planning; therefore, accurate tourism demand forecasting becomes vital. Artificial intelligence (AI) models such as neural networks and security violation report (SVR) have been used effectively in tourist demand forecasting as a result of the fast advancement of AI. This paper constructs a tourism demand forecasting model based on machine learning on the basis of the existing forecasting model research. The completed work is as follows: (1) It introduces a large number of domestic and foreign literatures on tourism volume forecasting and proposes the research content of this paper. (2) It is proposed to stack the long short-term memory- (LSTM-) based autoencoders deeply, by adopting a hierarchical greedy pretraining method to replace the random weight initialization method used in the deep network and combining this pretraining stage and fine-tuning network together to form the SAE-LSTM prediction model for improving the performance of deep learning models. (3) This paper uses the monthly search engine strength data of city A's monthly tourist volume and its related influencing factors as the data set; processes the data set to make the model adapt to the data input; uses mean absolute error (MAE), root mean square error (RMSE), MAPE, and other model evaluation indicators; and uses LSTM and the constructed SAE-LSTM model to conduct comparative experiments to predict the number of tourist arrivals in four years. The prediction results of the models proposed in this paper are better than those of the LSTM model. According to the experimental results, the superiority of the proposed LSTM-based unsupervised pretraining method is demonstrated.

## 1. Introduction

With the development of the times, tourism has become an important economic industry in today's world, and tourism has become an indispensable part of modern people's daily life. With the rapid development of the tourism industry, many other problems have arisen. Popular tourist attractions are overcrowded, causing damage to the environment and many safety incidents. The relevant management personnel lacked experience in emergency handling and could not handle it in a timely manner, and the scene was once chaotic. If the flow of people exceeds expectations and there is no effective management, it will bring about serious stampede incidents. For popular tourist attractions, people flow restriction measures and emergency plans should be formulated to improve risk prevention awareness. Many studies have been carried out in the academic community. Nowadays, in the information age, various situations spread rapidly, and once a safety accident occurs, it will spread rapidly. Even if corresponding measures are formulated, it is difficult to reduce the social impact, causing losses to tourist attractions, which is not conducive to long-term development [1–3]. Therefore, relevant personnel of tourist attractions should pay attention to the occurrence of safety accidents, formulate effective management systems and countermeasures, and cultivate awareness of prevention among all employees. In the process, whether it is the scenic spot manager or the relevant departments, it is necessary to clarify the prevention standards and build a perfect system to predict the tourist flow and prevent problems before they occur. While avoiding excessive tourist flow, it is also necessary to avoid the loss of tourism in the off-season, especially in hotels and transportation, which will cause waste of resources and affect the sustainable development of scenic spots [4, 5]. It can be seen that the development of the tourism industry is affected by many factors, which will cause seasonal and cyclical changes. It is necessary to pay attention to the timely and accurate judgment of the tourism volume, improve the utilization rate of resources, improve the management ability of scenic spots, and ensure that the tourism industry can form a sustainable development. In order to prevent various problems caused by excessive human flow, it is necessary to predict the passenger flow in advance, improve the carrying capacity of the scenic spot, and formulate effective preventive measures to avoid it, so as to improve the utilization rate of resources and evenly distribute the passenger flow. Therefore, research on the tourism industry must focus on the forecast of tourism volume, which can promote the simultaneous improvement of market value and academic value, and has attracted attention from all walks of life. Aiming at the problem of tourism demand forecasting, statistical methods are used for modeling, and good results have been achieved [6]. To begin, linear regression was employed to predict tourist demand. It was possible to develop a model for forecasting tourist demand by looking at the link between historical demand data and estimated model parameters. Because the cyclical variation in tourist demand is not taken into account, the inaccuracy in predicting tourism demand is rather substantial. Some researchers have proposed methods based on moving average, exponential smoothing, and other time series analysis techniques to address the shortcomings of the linear regression model; however, these techniques are still essentially linear modeling techniques, and as a result, their limitations are also obvious [7]. With the advancement of neural network research in recent years, some researchers have proposed a neural network-based tourism demand forecasting model, which is a nonlinear modelling method that can not only describe cyclical characteristics of tourism demand but also track time-varying travel demand and produce good travel demand forecast results.

The article "Design of Machine Learning Algorithm for Tourism Demand Prediction" was published in 2022. Journal: Comput Math Methods Med.

It is suggested that the SVR model be employed in tourist forecasting. SVR is a small sample forecasting issue modeling that has the strong forecasting performance of a neural network and can overcome the disadvantages of overfitting. The neural network needs a large number of tourist demand samples, and tourism demand is a small sample prediction issue; thus, the neural network is prone to overfitting during the learning phase, although the fitting accuracy is rather good. The capacity of deep learning in tourism prediction is demonstrated by a tourism prediction model based on LSTM and attention mechanism [8–10]. As a result, the paper's main research goal is to present a tourism volume forecasting model that will improve forecasting accuracy. The proposed model will enable the tourist department comprehend the passenger flow distribution in advance so that scientific decisions can be made, and the strategy will also save a lot of tourism resources, which has far-reaching practical implications.

The paper structures are as follows: Section 2 discusses the related work.  Section 3 defines the various methods.  Section 4 analyzes the experiment and analysis.  Section 5 concludes the article.

## 2. Related Work

Nowadays, the social economy is in a period of rapid development, and the proportion of tourism in the entire economic life is increasing. There is an urgent need to conduct more in-depth research on tourism volume forecasting. At present, after sorting out relevant literature, it is found that foreign research on tourism volume forecasting is mainly divided into three stages: traditional econometric model research, artificial intelligence model research, and hybrid model research, which have more accurate forecasting effects. The earliest traditional econometric model adopts the form of time series. Through long-term use, the model structure is relatively mature, focusing on the characteristics and variable parameters of the data associated with the model, which are determined by the changing trend and shape of the time series; then, through the analysis of the econometric model, the change of the target time series is determined. It can be seen that the observation object of the time series model is only the historical data of the predictor variable, so the data collection is simple, and the application cost is very low, but there is a certain deviation in the prediction result. For a long time in the past, time series models have been used in the forecast of tourism volume and have been popularized in many fields. The more famous one is the comprehensive autoregressive moving average model proposed by reference [11] in 1970. After that, the use of time series models made a breakthrough in 2000, and simple ARIMA models and SARIMA models were constructed, which were recognized and popularized by the academic community. Since the tourism measuring tool is greatly affected by the seasonality, the model can effectively grasp this feature and improve the prediction accuracy [6]. Many innovations were then carried out on this foundation. Reference [12] conducted extensive study on tourism volume forecasting, built a GARCH model using three multivariables, and examined the corresponding factors impacting tourism volume through real verification. Market demand is influenced by different types of markets. In addition, reference [13] analyzed and compared the forecast differences between the econometric models and analyzed the Indian tourism market through the forecast results obtained by the X-12-ARIMA model and the ARFIMA model. Also, typical is the traditional econometric model, which is also one of the more mature forecasting models. The core foundation of the traditional econometric model is statistics, which integrates the knowledge of various disciplines. Based on the mathematical model, the actual parameters are added to form a random setting form, and then, the relationship between variables and influencing factors is analyzed through the application of the model. At present, there are many forms of econometric methods in tourism volume forecasting, mainly including vector autoregressive model (VAR), autoregressive distributed lag model (ADLM), error correction model (ECM), and time-varying parameter (TVP) model, and all of them have been effectively applied [14–16]. Reference [17] used the VAR method to successfully predict the number of tourists in popular scenic spots in a certain region of France in recent years. Then, taking the characteristics of different countries as the analysis point, we got the conclusion that the country is the largest market in the future and then compared the actual state for verification and summarized the results that the VAR model can effectively predict the medium and long-term tourism volume. In addition, through extensive practical analysis, VAR models can be constructed more simply because they are mainly based on theoretical analysis. After that, the research of reference [18] introduced a new method, which led to the development of inbound tourism forecasting. Reference [19] carried out error analysis on the existing basis and optimized the prediction model, so that the British outbound tourism volume was effectively analyzed. With the continuous development of research methods, the academic community has gradually realized that due to the problems of time series, the previous prediction models often fail to achieve the expected results. To this end, artificial intelligence models have been proposed through a large number of innovations, and AI-based technology has been greatly developed [20, 21]. At the end of the last century, the concept of artificial neural network (ANN) was introduced into the tourism volume prediction model, which made the research greatly developed. In this regard, reference [22] summarizes the ANN model for tourism volume prediction and puts forward a conclusion that is superior to the traditional model through analysis. Reference [23] believes that the ANN model has great advantages in tourism volume forecasting. Compared with the traditional Naivel model, ES method, multiple regression, and other models, it has many characteristics, and the prediction results are more effective. Reference [24] optimizes on the basis of ANN, compares multiple prediction models after summarization, and obtains many rules and summarizes the multilayer perception prediction model. With the continuous research on tourism volume forecasting, the accuracy of tourism volume forecasting based on various models has been continuously improved, but the transparency of the model is low, so that users cannot understand the mechanism of the model and thus cannot gain the trust of users. It is of great significance to study the interpretability of tourism forecasting models, but at this stage, there is no or very little work focused on interpretable tourism demand forecasting [25–27]. Many machine learning models are widely used in time series forecasting. If the traditional ANN with shallow structure becomes too complex, for example, the network contains many layers and parameters; it is difficult to train. Deep neural networks (DNNs) have shown better performance than traditional neural networks in many time series forecasting applications. Deep learning can train DNNs with many hidden layers, and it is easy to learn features from raw data, so it is very popular in the field of machine learning.

The article "Design of Machine Learning Algorithm for Tourism Demand Prediction" was published in 2022. Journal: Comput Math Methods Med.

## 3. Method

This section discusses the AE-LSTM prediction model construction. They define the SAE-LSTM prediction model construction, and they evaluate the selection of model evaluation indicators.

### 3.1. AE-LSTM Prediction Model Construction

Here, LSTM network and autoencoders are examined. They analyze the LSTM-based autoencoder pretraining model construction.

#### 3.1.1. LSTM Network

RNN has been used to solve problems such as tourism demand predictions because it can simulate dependencies between sequence data through loops. However, because the neural network is in the process of forward transmission, the influence of the later time on the previous time diminishes as the later time passes, so it is unable to recall the long-term memory. LSTM not only has a loop learning unit inside the network but also through the design gate to collect longer and shorter states from the start unit to the last unit; the recall of long-term memory is superior to RNN. The design of LSTM can effectively deal with long-term memory.  Figure 1 shows the LSTM model used in this paper. LSTM can process time series data sequentially and use the output of the last time step to predict the output of a linear regression layer. The LSTM memory cell is controlled by three gates to sequence the messages passed, thereby accurately capturing long-term dependencies. The three gates are responsible for controlling the interaction between different memory cells. The function of the input gate is to control whether the input signal can modify the state of the memory cell, the forget gate controls whether to remember the previous state, and the output gate controls the output of the memory cell.

In each time step *T*, the hidden state *h*^*t*^ is updated by the input *x*^*t*^ at the same time, the previous state of the hidden layer is *h*^*t*−1^, the input gate is *i*^*t*^, the output gate is *o*^*t*^, the forget gate is *f*^*t*^, and the storage unit is *s*^*t*^; the relational equation is as follows:

(1) $$\begin{array}{c} i^{t}=\lambda \left(w^{i}x^{t}+v^{i}h^{t-1}+a^{i}\right), \end{array}$$

(2) $$\begin{array}{c} f^{t}=\lambda \left(w^{f}x^{t}+v^{f}h^{t-1}+a^{f}\right), \end{array}$$

(3) $$\begin{array}{c} o^{t}=\lambda \left(w^{o}x^{t}+v^{o}h^{t-1}+a^{o}\right), \end{array}$$

(4) $$\begin{array}{c} s^{t}=f^{t}\times s^{t-1}+i^{t}\times \tanh\left(w^{s}x^{t}+v^{s}h^{t-1}+a^{s},\right.\; \end{array}$$

(5) $$\begin{array}{c} h^{t}=o^{t}\times \tanh\left(s^{t}\right), \end{array}$$

where *w*, *v*, and *a* are model parameters, which are continuously learned during model training; *λ* and tanh are excitation functions, which are responsible for mapping the input of the neuron to the output; × represents the product of the corresponding position elements of the two matrices; and the linear regression layer is as follows:

(6) $$\begin{array}{c} {\bar{y}}_{i}=w^{r}h_{i}^{t}, \end{array}$$

where *w*^*r*^ is the weight parameter of the linear regression layer, and formula (6) is used to predict the output of the linear regression layer.

The article "Design of Machine Learning Algorithm for Tourism Demand Prediction" was published in 2022. Journal: Comput Math Methods Med.

#### 3.1.2. Autoencoders

Autoencoder (AE) is divided into three parts, namely, input layer, hidden layer, and output layer, and is an unsupervised learning algorithm. The autoencoder training process used in this paper is divided into two stages: the encoding stage compresses the input data, and the decoding stage reoutputs the compressed data. The autoencoder structure is shown in Figure 2.

Among them, given the unlabeled data set *x*_*n*_, *n* = 1, 2, ⋯, *N*, the two stages of the autoencoder used in this paper can be expressed as follows:

(7) $$\begin{array}{c} h_{x}=f\left(w_{1}x+a_{1}\right), \end{array}$$

(8) $$\begin{array}{c} x_{o}=g\left(w_{2}h_{x}+a_{2}\right), \end{array}$$

where *w*_1_ is the weight parameter from input to hidden neural layer, *w*_2_ is the weight parameter from hidden to output neural layer, *a*_1_ and *a*_2_ are the deviation vectors of input layer and hidden layer, respectively, encoding refers to from input to hidden neural layer conversion, decoding refers to the conversion from hidden to output neural layer, *f* is the encoding function, *g* is the decoding function, and *h*_*x*_ represents the hidden encoding layer vector calculated from the input vector *x*, where the relationship between the input vector *x* and the output vector *x*_*o*_ is shown as follows:

(9) $$\begin{array}{c} x_{o}\approx x. \end{array}$$

Among them, the autoencoder is learned through training to ensure that *x* and *x*_*o*_ are equal to achieve a compressed representation of *x*. Autoencoders are often used to extract nonlinear features.

#### 3.1.3. LSTM-Based Autoencoder Pretraining Model Construction

The forecasting problem of tourism demand is a time series forecasting problem. Based on RNN, it is more suitable for modeling time series data. This paper proposes a new structure based on LSTM and autoencoder, which can extract features from time series problems, and is to replace the encoding layer and decoding layer of the autoencoder with the LSTM network layer, so as to propose an LSTM-based autoencoder pretraining model, as shown in Figure 3.

The article "Design of Machine Learning Algorithm for Tourism Demand Prediction" was published in 2022. Journal: Comput Math Methods Med.

This paper proposes an LSTM-based autoencoder pretraining model, which consists of two LSTM layers, an LSTM encoding layer and an LSTM decoding layer, given an input sequence (*x*_1_, *x*_2_, ⋯, *x*_*n*_); the encoder accepts the input sequence and encodes it into the learned representation vector; then, the decoding layer takes this representation vector as input and tries to reconstruct the input sequence (*x*_*o*1_, *x*_*o*2_, ⋯, *x*_*on*_). This structure is an unsupervised learning algorithm.

### 3.2. SAE-LSTM Prediction Model Construction

This section examines the stacked autoencoders. They discuss the LSTM-based stacked autoencoder pretraining model construction. They analyze the SAE-LSTM prediction model construction.

#### 3.2.1. Stacked Autoencoders

Deep learning is a machine learning method based on data learning. Data features are extracted through multilayered nonlinear processing units. Each layer uses the output of the preceding layer as input, and the data is translated from the bottom layer to the top layer. Deep networks can learn more representations and better identify correlations between data by stacking layers on top of each other. Stacked autoencoders (SAE) essentially use the output of the hidden layer of the previous autoencoder as the input of the next autoencoder, which is composed of multiple autoencoders. Each autoencoder is utilized as a hidden layer, and many hidden layers are piled successively from the bottom to produce the stacked autoencoder deep network. In this structure, multiple autoencoders are stacked, and each autoencoder layer is trained so that the input error is locally optimal, and the output of the hidden layer is used as the input layer of the next autoencoder layer. A single autoencoder can learn a feature representation through the three-layer network of equation (10), such as the following:

(10) $$\begin{array}{c} x⟶H_{1}⟶x_{o}, \end{array}$$

(11) $$\begin{array}{c} H_{1}=f_{\mu }\left(x\right). \end{array}$$

The stacked autoencoder obtains *H*_1_ through the training of the first autoencoder and then uses *H*_1_ as the input to train the next autoencoder to obtain *H*_2_ and then continues to train this deep learning structure. That is, first train equation (10) to obtain the transformation of equation (12), and then, train equation (13) to obtain the transformation of equation (14), and finally, stack the SAE layer by layer.

(12) $$\begin{array}{c} x⟶H_{1}, \end{array}$$

(13) $$\begin{array}{c} H_{1}⟶H_{2}⟶H_{1}, \end{array}$$

(14) $$\begin{array}{c} H_{1}⟶H_{2}. \end{array}$$

#### 3.2.2. LSTM-Based Stacked Autoencoder Pretraining Model Construction

The progressive unsupervised pretrained stacked autoencoder can learn the features of the original data layer by layer, which is more suitable for complex features. Therefore, this paper proposes an LSTM-based stacked autoencoder pretraining model. The LSTM-based stacked autoencoder is also a greedy hierarchical pretraining, and its construction process is divided into the following three steps:

1. First train the first LSTM-based autoencoder; then, save its LSTM encoding layer and its learned network parameters, and use the first LSTM encoding layer as the input of the second LSTM-based autoencoder
2. In order to train an LSTM-based autoencoder, load and utilize the previously stored encoder layer to recreate the original input data, not the encoded input data. This allows the encoder to pick up on characteristics from the original data and improve its performance. Save the learned network parameters and the second LSTM-based encoding layer using the second LSTM-based encoding layer as an input to the third LSTM-based self-encoder
3. Load the two saved encoder layers, use them to encode the input twice, then continue to train the third LSTM-based autoencoder with the saved encoded version, thereby reconstructing the original input and saving the third LSTM-based autoencoder encoding layer and its learned network parameters. And so on, this model can also be generalized to more than three layers

The article "Design of Machine Learning Algorithm for Tourism Demand Prediction" was published in 2022. Journal: Comput Math Methods Med.

#### 3.2.3. SAE-LSTM Prediction Model Construction

The SAE-LSTM tourism volume prediction model is constructed using a stacked autoencoder based on LSTM to replace the random initialization of weights used in the LSTM network. Taking the training of three LSTM-based autoencoder stacks as an example, the SAE-LSTM model is divided into a pretraining stage and a fine-tuning stage, in which the three encoding layers and the optimized network parameters are saved in the pretraining stage. The fine-tuning stage is divided into two steps:

1. Using the three LSTM encoding layers and their learned network parameters saved in the pretraining stage
2. Add an output layer on top of the three hidden layers, which have only one node and is utilized to solve the tourism volume forecast problem

### 3.3. Selection of Model Evaluation Indicators

In order to evaluate the performance of the prediction model, this paper uses three evaluation indicators to evaluate the prediction effect. They are mean absolute error (MAE), root mean square error (RMSE), and mean absolute percentage error (MAPE). Given the predicted value *y*_*p*_ and the actual value *y* as follows:

(15) $$\begin{array}{c} y_{p}=\left\{y_{p1},y_{p2},\cdots ,y_{pn}\right\}, \end{array}$$

(16) $$\begin{array}{c} y=\left\{y_{1},y_{2},\cdots ,y_{n}\right\}. \end{array}$$

The three index equations are as follows:

(17) $$\begin{array}{c} \text{MAE}=\frac{1}{n}\overset{n}{\underset{i=1}{\sum }}\left|y_{pi}-y_{i}\right|, \end{array}$$

(18) $$\begin{array}{c} \text{RMSE}=\sqrt{\frac{1}{n}\overset{n}{\underset{i=1}{\sum }}{\left(y_{pi}-y_{i}\right)}^{2},} \end{array}$$

(19) $$\begin{array}{c} \text{MAPE}=\frac{1}{n}\overset{n}{\underset{i=1}{\sum }}\left|\frac{y_{pi}-y_{i}}{y_{i}}\right|, \end{array}$$

where MAE is a measure of the average magnitude of a set of errors, and it is the sum of the absolute values of the differences between *y* and *y*_*p*_ and then divided by the number of test samples; RMSE is a measure of the average magnitude of a set of errors, which is the square root of the average of the squared differences between *y* and *y*_*p*_; and MAPE is the mean of the absolute value of each error divided by *y*. The three indicator formulas are calculated by the predicted value and the actual value. The larger the three values, the larger the error.

The article "Design of Machine Learning Algorithm for Tourism Demand Prediction" was published in 2022. Journal: Comput Math Methods Med.

## 4. Experiment and Analysis

This section discusses the data preprocessing. They evaluate the experimental design and model parameter selection. They analyze the analysis of experimental results.

### 4.1. Data Preprocessing

Here, the data sources are defined. They examine the data preprocessing.

#### 4.1.1. Data Sources

The data set used in this paper is the monthly search engine strength data of the number of monthly passenger arrivals and tourism-related influencing factors in a region from January 2014 to December 2019, and the region is represented by city A. Among them, the monthly tourist arrivals are provided by the tourism bureau of the city government. The tourist arrivals collected from the DSEC website in this article are the tourist arrivals from the global market. The experimental data of this paper adopts the search engine strength data of 168 influencing factors related to tourism in city A, of which 38 monthly search engine data are from Baidu and 130 monthly search engine data are from Google. The influencing factors of the seven tourism categories are extended, and Table 1 lists some of the influencing factors used in the experimental data.

To sum up, the experimental data in this paper consists of the monthly search intensity of 168 tourism keywords and the arrivals of tourists in city A. This time series data is a list with ordered values.

#### 4.1.2. Data Preprocessing

*(1) Data Normalization*. Data normalization is the process of scaling data into a specific range. The data of city A is normalized using min-max normalization in this study, so that each characteristic is of the same order of magnitude. The conversion function used is shown as follows:

(20) $$\begin{array}{c} I^{*}=\frac{I-\min}{\max-\min}, \end{array}$$

where min and max are the minimum and maximum values of the sample data; min-max normalization can make the sample data fall within the [0, 1] interval.

*(2) Data Conversion*. The sliding window is a fixed-length data movement, one unit at a time; for example, January 2014 to December 2019 is a fixed-length data, the length of this window is 12, and this window is from left to right glide; assuming the data collection is on a monthly basis, the next window is not January 2015 to December 2015 but February 2014 to January 2015. The window slide travels one unit to the right at a time, and each window is always 12 inches in length. In other words, the time series data employed in this study is cyclical. The impact of data periodicity on forecasting difficulties can be reduced by using a sliding window to provide a fixed length for data conversion. The time series is made up of sequences that are ordered in chronological order. The data for this study is collected on a monthly basis. This paper converts the original data into time series data based on sliding windows. Given a time series *T* and a window of length 12, *T* = (*x*_1_, *x*_2_, ⋯, *x*_*n*_), *n* is 72, representing 72 months of data collected from January 2014 to December 2019; each *x* is also a 168-dimensional vector, representing the monthly search intensity of 168 tourism-related features. In this paper, the data is moved by the shift function of pandas. First, the time window is placed at the starting position of *T*, and then, the time window is moved one month backward with time, and then, the second month of *T* is used as the starting position, get the second data of length 12, and so on; there are a total of 60 data of length 12 *c*_1_, *c*_2_, ⋯, *c*_60_, where (*c*_1_ = *x*_1_, *x*_2_, ⋯, *x*_12_), (*c*_2_ = *x*_2_, *x*_3_, ⋯, *x*_13_). The converted data is as follows:

(21) $$\begin{array}{c} W_{\left(c\right)}=\left\{c_{i}\left|i=1,2,\cdots 60\right.\right\}. \end{array}$$

The second step of data conversion is to convert the sliding window-based city A time series data into supervised learning data to facilitate subsequent training of the model. The supervised learning data format consists of input and output, that is, predicting the output from the input. This article adds the actual passenger arrivals to city A in the next month on the basis of each *c*_*i*_.

The article "Design of Machine Learning Algorithm for Tourism Demand Prediction" was published in 2022. Journal: Comput Math Methods Med.

### 4.2. Experimental Design and Model Parameter Selection

Here, the experiment design phase is discussed, and the model parameter selection is evaluated.

#### 4.2.1. Experiment Design Phase

The specific experimental design phase is divided into three steps:

1. Process the city A data set, and then divide the processed data into training set, validation set, and test set. When predicting the 12-month tourism arrivals in 2016, the data sets of 2014 and 2015 are used as the training set, and the top 10% of the data are divided from the training set as the validation set, and then, the test set of this paper is the 12-month 2016 data set. When predicting the 12-month tourism arrivals in 2017, the first three years of data are used as the training set, the first 10% of the data are divided from the training set as the validation set, and then, the 2017 12-month data set is used as the test set, and so on to forecast the tourism volume from 2016 to 2019
2. Use the training set to train each model separately and predict the total amount of tourism for each model. The corresponding real tourist volume will be collected from the test set to produce new training data once the prediction model predicts the tourism volume for a month. Then, do the next step of training and prediction and so on to predict the number of tourists in city A from 2016 to 2019. And the hyperparameter involved in this paper is set based on past experience, and grid search is performed to perform brute force search, so as to obtain the best experimental results
3. Save the experimental results of each model and analyze the experimental results

#### 4.2.2. Model Parameter Selection

This paper uses the Keras deep learning framework to build the SAE-LSTM prediction model and builds the LSTM benchmark model for comparative experiments. This section describes the selection of model parameters during the experiment.

*(1) SAE-LSTM Prediction Model*. The construction process of the SAE-LSTM model used in this paper is the same as that in Section 3.2. For the SAE-LSTM model, it is divided into a pretraining stage and a fine-tuning stage. Regarding the preprocessing stage, the number of layers of the LSTM superimposed autoencoder is selected. In this paper, a trial and error method is used to predict the number of layers, and MAPE is used as the evaluation index. The specific experimental results are shown in Table 2.

It can be seen from Table 2 that the MAPE value of the SAE-LSTM model with more than three hidden layers is extremely high, which means that the error is very large; it shows that the high number of hidden layers will lead to overfitting. In order to avoid overfitting, the SAE-LSTM model with at most two hidden layers is used in the experiment. The SAE-LSTM of the two hidden layers is divided into a pretraining stage and a fine-tuning stage based on LSTM-based stacking autoencoders. The pretraining stage is the training of two LSTM-based autoencoders, thereby saving the two LSTM encoding layers and their trained parameters for the fine-tuning stage. The hyperparameters that need to be selected for the SAE-LSTM of the two hidden layers are the number of iterations epochs, the loss rate dropout, the number of units in the first coding layer lstm_unit1 in the pretraining stage, and the number of units in the second coding layer lstm_unit2. In this paper, grid search is used to obtain the optimal hyperparameter set of the SAE-LSTM prediction model of two hidden layers. Through grid search, the epochs are {200, 400, 500}, the dropout is {0.01, 0.2, 0.3}, lstm_unit1 is {56, 64, 128}, and lstm_unit2 is {32, 48, 64}.

*(2) LSTM Model*. In this paper, the LSTM model is selected as the benchmark model for the experiment. The LSTM model is introduced in Section 3.1.1. For the benchmark model, parameters are also selected from grid search.

The article "Design of Machine Learning Algorithm for Tourism Demand Prediction" was published in 2022. Journal: Comput Math Methods Med.

### 4.3. Analysis of Experimental Results

In this paper, the SAE-LSTM model and the LSTM model are used to conduct experiments on the city A data set. In order to avoid overfitting, SAE-LSTM only selects the two optimal hidden layers in training. And three model evaluation indicators MAE, RMSE, and MAPE are used to predict the accuracy. The tourist arrivals of the data set are tourists from city A around the world, and the tourist arrivals of this type fluctuate periodically. This paper uses this data set for experiments, and the experimental results are shown in Figures 4–6.

It can be seen from Figures 4–6 that the evaluation index value of two-layer SAE-LSTM is smaller than that of LSTM for 4 consecutive years. So it can be concluded that the SAE-LSTM prediction accuracy proposed in this paper outperforms the LSTM model in all performance measures. The experimental results show that the pretraining method of superimposing LSTM in the way of autoencoder has better performance than random initialization of LSTM weights, which proves that the proposed unsupervised pretraining method based on LSTM can replace the random weight initialization method used in deep networks. The feasibility of using this method to fine-tune the network improves the performance of the tourism volume prediction model.

## 5. Conclusion

With the increase in the number of tourists, the tourism industry has also tackled new challenges. The perishable nature of tourism products causes waste in the tourism industry, unsold rooms and air tickets cannot be stored, and the number of tourists and the distribution of tourism resources in many tourist attractions are gradually uneven, and accurate forecast of tourism volume can enable the number of tourism practitioners to allocate appropriate tourism resources to meet the tourism demand and reduce the waste of resources, and government agencies and tourism enterprises can use the accurate tourism volume forecast results to invest in basic measures and formulate tourism-related policies. The accuracy of tourism demand forecasting is critical, and this research presents a deep learning approach to help with that. This paper's primary work is summarized as follows:

1. Since recurrent networks are more suitable for modeling time series data, this paper first proposes to stack LSTM-based autoencoders deeply and replace the deep network with a layered greedy pretraining method. The SAE-LSTM prediction model, which is based on the suggested random weight initialization method, combines this pretraining stage and fine-tuning network to improve the performance of the deep learning model and obtain superior prediction results
2. In order to prove the effectiveness of the proposed deep learning model, this paper uses the monthly search engine intensity data of city A's monthly visitor volume and its related influencing factors from January 2014 to December 2019 as a data set to process the data set; adapts the model to the data input; uses MAE, RMSE, and MAPE model assessment indicators; and performs comparison tests using LSTM and the developed SAE-LSTM model to forecast the number of tourists in four years. The prediction results of the model proposed in this paper are all better than the LSTM model. According to the experimental results, the superiority of the proposed LSTM-based unsupervised pretraining method is demonstrated

The article "Design of Machine Learning Algorithm for Tourism Demand Prediction" was published in 2022. Journal: Comput Math Methods Med.

## Figures and Tables

**Figure 1:** LSTM model.

**Figure 2:** Autoencoder structure.

**Figure 3:** LSTM-based autoencoder pretrained model.

**Figure 4:** MAPE comparison of the two models.

**Figure 5:** MAE comparison of the two models.

**Figure 6:** RMSE comparison of the two models.

**Table 1:** Influencing factors of tourism in city A.

Travel category	Influencing factors
Dining	Gourmet, snack, famous restaurant
Lodging	Hotels, homestay, city bus
Tour	Tourist volume, tourism index
Clothing	Weather, air quality
Shopping	Shopping mall, shopping street
Recreation	Bar, concert
Transportation	Yacht, motorboat

**Table 2:** SAE-LSTM experimental results with different number of hidden layers.

Number of hidden layers	MAPE
1	3.158
2	3.125
3	3.388
4	6.753
5	6.923

## Data Availability

The data sets used during the current study are available from the corresponding author on reasonable request.
